RETRACTED

# Smartphone-Based mHealth and Internet of Things for Diabetes Control and Self-Management

**DOI:** 10.1155/2021/2116647

**Published:** 2021-10-16

**Authors:** Abolfazl Mehbodniya, A. Suresh Kumar, Kantilal Pitambar Rane, Komal Kumar Bhatia, Bhupesh Kumar Singh

**Affiliations:** ^1^Kuwait College of Science and Technology (KCST), Doha Area, 7^th^ Ring Road, Kuwait; ^2^School of Computing Science and Engineering, Galgotias University, Greater Noida, Utter Pradesh, India; ^3^KCEs College of Engineering and Management, Jalgaon, Maharashtra 425001, India; ^4^Department of Computer Engineering, J.C. Bose University of Science & Technology, Faridabad, India; ^5^Arba Minch Institute of Technology, Arba Minch University, Arba Minch, Ethiopia

## Abstract

In patients with chronic diseases condition, mobile health monitoring facility proves to play a significant role in providing significant assistance toward personal management. This research examined the use of smartphones by diabetes patients and their intentions to apply them for self-care and monitoring as well as management. This cross-sectional survey-based study was conducted in Jul-Aug 2021 with 200 diabetic patients (especially type 2) who were visiting specialized clinics and hospitals of Gujrat state, India. A validated questionnaire survey was designed to collect data, which included questions about demographics, information pertaining to other, use of cellphones, the Internet, and the intention to implement smartphones for diabetes monitoring, self-care, and self-management. A highest number of studied participants have mobile phone (97.5%) and smartphones (87%) and access the Internet on daily basis (83.5%). Younger participants were more inclined to use smartphone apps and have also shown more interest for continuous use in the future (*p* < 0.01). The majority of participants used apps for nutritional planning (85.5%), to monitor glucose control (76.5%), and for scheduling of diabetes appointments on the calendar (90.5%). Recommendations to use mobile app by doctors or healthcare profession were reported by 20.5% of the participants and attitude and future intention to use mobile apps were reported by the majority of participants. The majority of type 2 diabetes patients choose to use their cellphones and the internet or mobile phone reminder system for medication as well as to plan their diets, monitor their blood sugar levels, and communicate with their doctors. The findings of this research can be used to develop strategies and implement mHealth-based therapies to assist patients with type 2 diabetes to efficiently manage their health and might contribute to reducing patients' out-of-pocket expenditure as well as reducing disability-adjusted life years (DAILY) attributed by DM.

RETRACTED

## 1. Introduction

The incidences of diabetes are increasing globally. As per the International Diabetes Federation (IDF), the worldwide prevalence of DM, among the individuals that fall in the age group of 20 to 79, that was 9.3% in 2019 with projection of 10.9% roughly about 700 million in 2045 to be, which means an increased burden of 51% [1]. Even though there is improvement in the effective screening, diagnosis, and treatment, the elevated incidence of noncommunicable diseases such as DM and hypertension continues to be one of the major risk factors for morbidity and mortality among both developed and developing countries [2]. Diabetes stands seventh in being a causative factor for mortality around the world [3, 4] and has been associated with various complications, including cardiovascular diseases (CVD), cerebrovascular, retinopathy, nephropathy, amputation, and depression [5]. Diabetes is considered an incurable condition; however, it can be controlled by altering daily habits, i.e., lifestyle and self-management. Diabetes education empowers individual with DM to be more inclined toward their personal self-care and thus helps to procrastinate its future complications [6].

One of the first steps toward equipping diabetes patients with improved disease control is to enforce self-management, self-care, and monitoring behaviors [7]. However, many diabetes patients face a number of obstacles to effective self-monitoring, care, and management in the areas of blood glucose control, visceral fat, body fat and weight, hypertension control, and nutrition [8, 9]. Given the rise in the incidence of diabetes, the need of self-monitoring, care, and practical self-management techniques for diabetic patients should be considered [10]. Mobile-assisted educational interventions have the ability to shift nursing and treatment attention away from hospitals and onto the individual's everyday life [11].

Treatment failure is associated with reduced treatment benefits and can have a negative financial burden on both individual patients and the society at large [12]. Cost for management of DM includes intangible cost, direct cost, and indirect cost [13]. We know that finance of DM is uninsured and thus increased out-of-pocket (OOP) expenditure can lead toward poor medication adherence, thus resulting in a suboptimal benefit of treatment and leading to poor health outcomes [13]. Thus, an IoT-based DM management platform not only has potential to improve health outcomes, but it has also been shown to lower health-related costs and out-of-pocket expenses by reducing the number of clinic visits [14, 15].

RETRACTED

With the introduction of cellphones, IoT-based interventions, such as mobile phone-based medical health technology (mHealth) [16], are thought to have a bright future for promoting self-care, monitoring, and self-management via an inbuilt feature that aids in improving behavior change support systems (such as providing information, training, and reminders) [17]. mHealth refers to the use of devices such as smartphones or other wireless technologies to enhance health-related services [18]. It is one of the arms of electronic health (eHealth) [19].

Electronic health technologies, such as texting patients or service providers and smartphone-based applications (apps), aid in developing future opportunities for improved communication between patients and physicians, nurses, and other healthcare personnel [20]. The user-friendly design and mobility of mHealth technologies are only a few of the possible benefits for illness screening, early prediction, diagnosis, and fast treatment, therefore avoiding disease's negative effects and increasing cost-effective access to health services [21]. Despite its potential beneficial implications and growing interest, eHealth, particularly mHealth, has not been widely implemented [22]. The patient's individual positive attitude toward adopting mHealth treatments is one of the main variables that plays an essential part in their effective completion; nevertheless, there is a big gap in fully comprehending the patient's attitude toward this aspect [23]. There are few reviews of literature as well as research studies that have already investigated the use of mobile health that shows a huge potential in promoting self-management among patients with chronic diseases. There are many applications available in market such as glucose buddy, Intelligent Diabetes Management (IDM), BlueStar, Dbees, Bant2 Diabetes Interactive Diary (DID), GoCARB, Diabeo, D-Partner, Diabetes Pal, Diabetes Manager, and Diabetes Diary that have shown a promising improvement toward management of DM and VoiceDiab [24].

However, there are few research articles that highlights 3 major barriers amongst the nonapp users: there are certain reasons due to which they have a feeling that they do not need any app; firstly, it is due to lack of awareness about the available management apps; secondly, it is due to not having previously considered taking help of apps for self-management. Apart from this, participants frequently stated that their diabetes was not severe enough to warrant an app or that their existing traditional way of treatment was adequate and that an app would not enhance their situation [25].

Mobile phone penetration in rural India is high and this provides us a huge opportunity to instrument mobile phones in delivering diabetes education messages.

RETRACTED

The goal of the study was to determine the prevalence of patients using mobile phones and the internet for diabetes control and management, as well as their knowledge, attitude, and intention toward using mobile/smartphone apps for diabetes control and self-management, and to show the relationship between demographic parameters and knowledge, attitude, and intention to use mobile/smartphone apps for diabetes control and self-management.

## 2. Methods

### 2.1. Study Setup

In 2021, 200 individuals with type 2 diabetes visited a specialized diabetic clinic or one of two endocrinology and metabolism experts in the north of Gujarat for this cross-sectional research (India). A validated questionnaire was used to gather data, which included questions on demographics, illness information, usage of mobile phones, smartphones, and the Internet, and the desire to utilize mobile phones for diabetes self-management.

The study period was from July 2021 to August 2021 (2 months). Universal random sampling was used. We conducted a cross‐sectional study from several clinics and hospitals among patients suffering from type II diabetes. The design of the survey was adjusted who used mobile and smartphone app for diabetes control as well as for its management. Questions about diabetes status, demographic factors, type of diabetes, medication usage, self-care behavior, blood glucose level, perceived confidence in self-management competence, and perceived metabolic control were included in the Gujarati and English versions of the questionnaire. Chronic and acute health issues, the length of diabetes, medicine intake (medication practices) for diabetics, and the most recent glucose readings were all part of the health status. In addition, participants were asked about their smartphone ownership, kind of smartphone, and diabetes smartphone app usage. The use of a mobile phone includes the amount of time spent on the phone and the use of the phone for health information, diabetes awareness, and behaviors. A modified licensed version of the Summary of Diabetes Self-care Activities Questionnaire (SDSCA) [26] was used to assess self-care behavior as this questionnaire is a brief still promising and valid self-report measure of diabetes self-management which is a useful tool both for research as well as practice [26].  Figure 1 shows the work flow of the present research.

### 2.2. Ethical Standards

Ethical approval was obtained from the Institutional ethical committee (IEC code no. 236/2021). The survey was carried out in accordance with the institute's ethical standards. A written as well as an oral explanation was provided before to the poll to educate all respondents of the survey's anonymity. They were also told that taking part in the survey is completely voluntary, that their replies would be kept private, and that if they are uncomfortable, they may opt out at any time. Before taking part in the poll, respondents were also asked to provide their consent.

RETRACTED

### 2.3. Questionnaire Tool

The data was obtained using a modified questionnaire prepared by Dobson et al. study [27] revised based on the study's goals and the opinions of a health information management specialist, a medical informatics expert, and an endocrinologist, who all agreed that it was face-valid. Experts checked the questionnaire's content validity. The item content validity, such as relevance, clarity, and comprehensiveness of the complete instrument, was rated using a Likert scale (from unfavorable = 1 to fully favorable = 5) based on the views provided by the listed experts.

Following validation, the questionnaire included a few more items, such as demographic information, illness information, mobile phone and Internet use, intent to use mobile phone applications to control diabetes, and general explanations.

Gender, age, location of residence, education, and employment were among the demographic questions. They were also questioned about their diabetes care practices and challenges.

Choosing an acceptable diet, getting enough exercise, communicating with the doctor and other healthcare professionals, maintaining a positive connection with friends and family, keeping a blood glucose diary, and setting clear and specific diabetes management objectives were among the challenges.

Participants were given a few broad questions on their usage of mobile phones and the Internet, such as if they had a mobile phone or the Internet access, and how long they used it for. Aside from that, the participants were asked about their most common usage of mobile phones. Aside from that, the participants' intentions and attitudes regarding utilizing the Internet and mobile phones to manage diabetes were examined, and they were questioned about any services they needed to manage their illness. “For me, utilizing smartphone applications for self-management may be a, fun, excellent idea, easy, thrilling, useful, and inexpensive,” according to seven questions. These questions use a five-point Likert scale, with one being extremely terrible and five being very good.

A question based on a 5-point Likert scale (from no intention = 1 to very high intention = 5) was also asked of participants regarding their intention to utilize apps in the future.

RETRACTED

### 2.4. Data Collection

The researcher went to the diabetic clinic and specialist's offices to gather information. The researcher gave the patients an overview of the study's goals and instructions on how to fill out the questionnaire. The confidentiality of data and signed written informed consents were ensured following the survey. The questionnaires were completed by the patients in the presence of the researcher so that any misunderstandings could be resolved. A total of 287 type II diabetes patients were found at the clinic and doctor's offices, with 200 agreeing to complete the questionnaire, resulting in a response rate of approximately 67 percent. The surveys were completed by all 200 participants.

### 2.5. Data Analysis

The Pearson Correlation analysis produces a sample correlation coefficient, which evaluates a linear relationship among the variables in population. Statistical significance was set at *p* < 0.05. Further, post hoc test analysis was used for finding a significant correlation with knowledge and intention to apply smartphone apps in the future and also accept recommendation by healthcare providers to use these smartphone apps.

## 3. Results

The investigator double-checked all of the replies to ensure data quality. The replies that were received in their whole were discarded. Data from the lime survey was exported to Microsoft Excel when it was completed. Analytical statistics SPSS version 20.0 was used to analyze the data. A descriptive statistic was used, as well as post hoc testing. First, the proportion and frequency of demographic data, as well as the usage and intention to use mobile phones and the Internet by participants, as well as self-management issues, were identified. The overall attitude score was calculated by adding the values of attitude scales and calculating their mean and standard deviation. One question was used to establish the intention score. Based on the information of weight (kg) and height (m), the body mass index (BMI) was calculated (cm). Pearson correlation analysis was used to examine the connections between demographic information and attitude, as well as intention and confidence. The Pearson Correlation analysis produced a sample correlation coefficient, which evaluates a linear relationship among the variables in population. Statistical significance was set at *p* < 0.05. Further, post hoc test analysis was used for finding a significant correlation with knowledge and intention to apply smartphone apps in the future and also accept recommendation by healthcare providers to use these smartphone apps.

Figure 2 shows demographic profile and disease related information. Out of 200 patients, 45 patients were women and the maximum number of studied participants (40%) belonged to age group of 50–60 years. The majority of participants were graduate (54%, *N* = 108) and lived in the urban cities (89%). Ninety-five participants suffered from other chronic conditions; out of them 28 had hypertension, 11 have cardiovascular problems, and 19 had respiratory problems. The rest of them have other diseases including cancer, thyroid, kidney, gastric, and neurological issues. The male participants' BMI was 32.4 ± 5.1 which was categorized under Obesity Class 1 [28] and BMI of female participants was classified as under “preobesity” title.

RETRACTED

The participants' usage of mobile phones and the Internet, as well as their desire to use them to control their diabetes, is summarized in Table 1. Out of 200 studied participants, only 5 participants did not have mobile phones and 87% (*N* = 174) have smartphone and 83.5% had daily access to the Internet. On average, 74% (*N* = 148) of the participants spent 2.5 hours per day using mobile phones and the Internet (53.5%, *N* = 107). The studied participants mainly used their mobile phone to communicate with relatives and friends (84.3%) and obtain information on the Internet (44.1%). They used their phones the lesser to send and receives emails (8.1%), as well as to shop online (12.2%). The majority of participants utilized their mobile phones and the internet to dietary planning (85.5%), monitoring blood glucose and other clinical data (76.5%), and scheduling diabetes appointments on calendar (90.5%). The cumulative self-care for diabetes control and management revealed that the application of modern technology among both genders found significant especially for usage of mobile phone and smartphone. Use of text message reminder for diabetic self-management also showed significant correlation among male and female participants. Other parameters did not show significant association for both genders (Table 1).

Table 2 shows the participants' knowledge, attitudes, and intentions about the use of mobile/smartphone apps for diabetes self-management and control. One-third of the participants stated that they intended to use apps for diabetes control in the future and (66.6%) and 69 (34.5%) participants reported that they were 61%–80% confident they would use apps for self-controlling of diabetes. However, recommendations by doctors or healthcare professionals were reported by 20.5% (*N* = 41) of the studied participants. Cost-effectiveness also bothered 29.5% (*N* = 59) of the participants. Potential technical and regulatory issues reported among 37% (*N* = 74) of the studied participants.

Table 3 displays correlation between demographic parameter and knowledge, attitude, and intention to utilize mobile phone apps for the diabetes and control and self-management. Gender classification had no significant correlation with knowledge, attitude, and intention to use the Internet and smartphone apps for diabetes self-control and management. Younger participants (>30–49 years) showed significant association for all three psychological parameters and confidence and follow healthcare professions' recommendation to use smartphone apps. Post hoc test analysis revealed that the higher education level (graduate, *p* < 0.001 and post graduate,*p* < 0.003) had higher significant correlation with knowledge and intention to apply smartphone apps in the future and also they accept recommendation by healthcare providers to use these smartphone apps. Occurrence of length of diabetes (for short duration) had poor attitude and intention to use phone apps among older age (>60 years), less educated (<10^th^ standard), and semiurban participants. On the other hand, the mobile Internet used was significantly associated with those who had diabetes for a longer time (*p* < 0.05).

RETRACTED

According to the findings, 183 (91.5%) of the participants answered that if they were unable to utilize mobile phones for self-management, and they would like assistance from other family members (e.g., husband and children). In addition, 125 (62.5%) participants expressed an interest in participating in future research examining the impact of using apps in diabetes management.

Figure 3 shows the output associated with the intention of the studied participants to use mobile phone app in control and self-management of diabetes. The majority of the participants need app to make immediate contact with their physician or doctor (98.9%) followed by the contact with other healthcare providers (84.6%). The least number of participants was opted for improvement in physical activity and quality of life (QoL).

## 4. Discussion

Many studies have found that employing mobile phone technology improves glycemic control significantly across the globe [24]. The development of mobile technologies and smartphone apps for diabetes prevention can be utilized as a paradigm for translational and implementation research. The main finding of the study revealed that more than 95% use mobile phone and only around 16% participants did not use the internet on daily basis. Majority of them used mobile app for the nutritional planning and monitoring of blood glucose and to make contact with health providers. These findings corroborate with Rangraz Jeddi et al.'s study who conducted cross-sectional study on 218 patients of type II diabetes [29]. In our study, young age group participants (>30–60 years) were positively associated with self-care attitude, knowledge, and future intention to use mobile app [30]; this finding is similar to Husted et al.'s study on smartphone app usage for diabetes by young participants [30]. Younger diabetes patients were more interested in utilizing apps and had a greater desire and confidence in doing so in the future. Diabetic patients with a higher education (graduate) had a more favorable attitude toward and confidence in using apps, and they used their phones and the internet more frequently [31, 32]. These findings might be explained by the fact that patients with a higher level of education have better reasoning and critical thinking abilities than others, resulting in greater judgement and trust in mobile health devices.

RETRACTED

On the other hand, to make contact with other diabetic patients was limited to only 66 participants and the barrier for limited number of participants assumed that they exclusively use it for monitoring of blood glucose and dietary planning.  Figure 4 shows the factors influencing the likelihood of the app. The result of this study was compared to other studies which also showed no significant difference reported between gender and attitude, knowledge, and intention to use app in the future, self-assurance in using smartphone apps, and also daily use of the internet and mobile phones [29]. Further, studied participants' knowledge, attitude, and other aspects toward practice of smartphone apps for the diabetes control and management showed more score values for cost-effectiveness, attitude, and future intention toward usage of app for the diabetes control. These criteria also showed similarity with Dobson and Hall's study, who also found significant correlation association between positive attitude and intentions toward using assistive technologies in self-management of diabetes [27]. The analysis for intention to use smartphone app revealed that the studied participants were more concerned with contacting their doctor and other healthcare professionals such as dietician and nurse. These findings were similar to Murlidharan et al.'s study on mobile heath technology for the prevention of type II diabetes [14]. Hussein et al. found that continuous and tailored support and contact with a diabetes educator and a physician via SMS text messaging reduced HbA1c by 1.16 percent in type 2 diabetes patients [33]. Glycemic control has improved in studies using SMS technology based on knowledge, attitude, practice, self-efficacy, and motivation [34, 35].

The amount of information gathered on current patterns of everyday technology use and self-management technology use, as well as self-efficacy and willingness to utilize these technologies for diabetes-related goals, may be used to guide future diabetes self-management technology research and development. Another highlight of this study was the use of in-person sampling (rather than online sampling), which minimized bias in technological choices.

RETRACTED

Here, we added a diagram (Figure 3) which summarizes the factors that influence app use and is based on a modified version of the Health Belief Model and the Health Information Technology Acceptance Model (HITAM). The combination of these frameworks provides an excellent theoretical foundation for study into mobile phone app user experience [27, 36].  Figure 5 shows the overview of mHealth intervention model work for management of not only individuals with DM but such a platform can be used by pre-DM (i.e., those with border line of DM) to avert DM. This help application developers to improve or modify their app toward more user-friendly and increase competence and further to improve their self-reported management deficits.

## 5. Conclusion

Finally, the majority of type 2 diabetes patients are willing to use their cellphones and the internet to plan their daily meals, monitor their blood glucose levels, and communicate with their doctors/consultants. This work adds to our understanding of how to design and execute mHealth-based treatments to improve diabetes self-management. A significant result is the need of healthcare practitioners being aware of apps as a self-management option and participating in their use to support improved patient outcomes and education. Smartphone or mobile phone usage among patients with diabetes mellitus is significantly sizeable in India. The participants welcome the use of mobile/smartphones to enhance their health practices and it requires no significant additional costs. Smartphones have potential application to be used to send reminders for clinic visits and to improve adherence to medication among patients with diabetes in urban India. The findings could help application developers improve the design and usability of their apps. These findings are crucial for general practitioners, nurse practitioners, and allied health professionals who may integrate apps into a holistic care strategy that considers techniques outside the clinical environment, given that self-management is a substantial element in glycemic control. As this mHealth platform helps in self-management, thus it seems to have huge potential in reducing patients' out-of-pocket expenditure as well as reducing disability-adjusted life years (DAILY) attributed by DM. Major limitation of this study is the sample size that was kept constrained due to the pandemic, so more research is needed to look into the perspective of health experts when it comes to app usage recommendations.

RETRACTED

## Figures and Tables

**Figure 1:** Block diagram of work flow.

**Figure 2:** Demographic and disease details of studied participants (*n* = 200).

**Figure 3:** Frequency percentage of participants' aim to use mobile/smartphone app in self-management of diabetes.

**Figure 4:** Modified diagram of factors that influence the likelihood of app use [25].

**Figure 5:** Overview of mHealth intervention for DM.

**Table 1:** Prevalence of mobile phones and the Internet used by the studied participants for the diabetes control and further management (*N* = 200).

Questions		Frequency (percentage)			Difference (*p* value)
		Yes	No	Unknown	
Application of modern technology	Usage of mobile phone	195 (97.5%)	5 (2.5%)	—	0.006^*∗*^
	Usage of smartphone	174 (87.0%)	26 (13.0%)	—	0.0001^*∗*^
	Access to the Internet on a daily basis	167 (83.5%)	33 (16.5%)	—	0.561
Inclination of using a mobile phone and the Internet to manage diabetes	Nutritional (dietary) planning	171 (85.5%)	26 (13.0%)	3 (1.5%)	0.312
	Monitoring blood glucose and other parameters	153 (76.5%)	38 (19.0%)	9 (4.5%)	0.213
	To make contact with specialist	124 (62.0%)	69 (34.5%)	7 (3.5%)	0.456
	Utilizing text messages as a diabetic self-management reminder	134 (67.0%)	55 (27.5%)	11 (5.5%)	0.001^*∗*^
	Listing of diabetes appointments on the calendar	181 (90.5%)	15 (7.5%)	4 (2.0%)	0.126
	Organization and scheduling of physical activity	139 (69.5%)	35 (17.5%)	26 (13.0%)	
	To make contact with other healthcare provider (nurse and nutritionist)	98 (49.0%)	67 (335%)	35 (17.5%)	0.489
	Contacting with other diabetic patients	66 (33.0%)	52 (26.0%)	82 (41.0%)	0.219

Self-care for diabetes control and management differences among male and female participants (^*∗*^ statistically significant).

**Table 2:** Participants' knowledge, attitude, and other factors toward usage of smartphone apps for the diabetes control and management (rated 1–5).

Questions	Mean ± SD (out of 5)
Attitude toward usage of app for the diabetes control	4.2 ± 0.6
Knowledge toward usage of app for the diabetes control	3.8 ± 0.7
Intention of studied participants to use apps for diabetes control in the future	4.3 ± 0.5
Recommendation by healthcare profession to use app for self-management of diabetes	3.6 ± 0.4
Lack of acceptance and doubt about smartphone apps for the diabetes control	4.5 ± 0.7
Cost-effectiveness	4.6 ± 0.5
Potential technical and regulatory issues	4.1 ± 0.3

**Table 3:** Correlation between participants' demographic profile, attitude, intention, and other parameters in association with the use of smartphone apps for diabetes self-control and management.

Demographic variables	Attitude	Knowledge	Intention (for future use)	Recommendation by healthcare provider	Other	Mobile and internet use
Age	−0.538^*∗∗*^	−0.291^*∗*^	−0.489^*∗∗*^	0.190	0.102	−0.350^*∗*^
Gender	0.012	0.034	0.094	−0.89	0.067	0.008
Education	0.357^*∗∗*^	0.581^*∗∗*^	0.431^*∗∗*^	0.090	−0.075	0.182^*∗*^
Occupation	−0.167^*∗*^	0.213^*∗*^	0.267^*∗∗*^	−0.086	0.148^*∗*^	−0.412^*∗∗*^
Occurrence of length of diabetes	−0.158^*∗*^	-0.321^*∗*^	0.225^*∗∗*^	−0.098	0.290^*∗*^	0.146^*∗*^

Correlation significance level at ^*∗*^*p* < 0.05 and ^*∗∗*^*p* < 0.01. Other parameters include lack of acceptance, cost-effectiveness, and potential technical and regulatory issues.

RETRACTED

## Data Availability

Data will be made available on request.

## Abbreviations

IoT: Internet of Things
DM: Diabetes mellitus
DAILY: Disability-adjusted life years
QoL: Quality of life
HITAM: Health Information Technology Acceptance Model
mHealth: Mobile health
IDF: International Diabetes Federation
CVD: Cardiovascular diseases
eHealth: Electronic health
DID: Diabetes Interactive Diary
SDSCA: Summary of Diabetes Self-Care Activities
BMI: Body mass index
m: Meter
cm: Centimeter
Kg: Kilogram
SD: Standard deviation.
